The article "Toll-Like Receptor 4 Exacerbates Mycoplasma pneumoniaevia Promoting Transcription Factor EB-Mediated Autophagy" was published in 2022. Journal: Contrast Media Mol Imaging.

# Toll-Like Receptor 4 Exacerbates *Mycoplasma pneumoniae*via Promoting Transcription Factor EB-Mediated Autophagy

**DOI:** 10.1155/2022/3357694

**Published:** 2022-07-31

**Authors:** Yan Liu, Jing Li, Xianfeng Lu, Shuangping Zhen, Jing Huo

**Affiliations:** Pediatrics Department, Shanxi Provincial People's Hospital, Taiyuan, Shanxi 030014, China

## Abstract

*Mycoplasma pneumoniae* (*M. pneumoniae*) is the most common cause of community-acquired pneumonia. Toll-like receptors (TLRs) play an essential role in pneumonia. The purpose of this study was to investigate the roles of TLR4 in *M. pneumoniae*. Mice were administrated with 100 *μ*l (1 × 107 ccu/ml) of *M. pneumoniae*. HE staining was applied for histological analysis. The protein expression was determined by western blot. The cytokine level was detected by ELISA. The results showed that TLR4-deficient mice were protected from *M. pneumoniae*. However, downregulation of TLR4 inhibited inflammatory response and autophagy. Moreover, transcription factor EB (TFEB) participated in *M. pneumoniae*-induced inflammatory response and autophagy, while knockdown of TLR4 downregulated TFEB and its nuclear translocation.

## 1. Introduction

*Mycoplasma pneumoniae* (*M*. *pneumoniae*) is an essential cause of community-acquired pneumonia [1]. The outbreaks of *M*. *pneumoniae* promote the progression of chronic and acute airway diseases, such as asthma [2]. Despite its self-limited and benign properties, *M*. *pneumoniae* is a public concern for the emerging antibiotic resistance [3]. Moreover, the outstanding side effects of *M*. *pneumoniae* therapies, such as fever, offset clinical results for its association with various complications (cytotoxicity, membrane fusion damage, invasive damage, toxic damage, DNA damage, autophagy, and inflammation) [4]. Therefore, to investigate an efficient therapy for *M*. *pneumoniae* is of vital importance.

Mycoplasmas induce the release of membrane-bound lipoproteins, which promotes the survival of bacteria [5]. Moreover, bacterial lipoproteins function as pathogenic substances to activate inflammatory responses via their recognition receptors [6]. For instance, *M*. *pneumoniae* increases the release of lipoproteins, which promotes inflammatory response via activating toll-like receptors (TLRs) [7]. TLRs are central pattern recognition receptors, which collectively participate in early recognition and the global and local immune response of the host to invading microbes [8]. TLRs recognize bacterial components, such as lipopolysaccharide (LPS), fibroblast-stimulating lipopeptide-1 (FSL-1), lipoarabinomannan, and zymosan, which increases the susceptibility of human hosts to various respiratory diseases [9–11]. TLR4, as a member of TLRs, plays a critical role in modulating immune responses to various molecular structures of microbes [12]. LPS-induced upregulation of TLR4 promotes *M*. *pneumoniae* infection [13]. Moreover, the activation of TLR4 signaling stimulates immune response and autophagy and exacerbates *M*. *pneumoniae* [14]. However, the potential roles of TLR4 in *M*. *pneumoniae* have not been fully elucidated.

In this study, we investigated the potential roles of TLR4 in *M*. *pneumoniae* and the underlying mechanisms. *M*. *pneumoniae*-induced overexpression of TLR4 contributed to inflammation response and promoted the transcriptional activity of TFEB, which further promoted lipid-induced autophagosome formation and evoked a proinflammatory response. Hence, the TLR4/TFEB axis may form a feedback loop to promote the release of proinflammatory cytokines.

## 2. Materials and Methods

### 2.1. *M*. *pneumoniae* Culture

*M. pneumoniae* strain M129 was consecutively cultured in Hayflick medium containing PPLO broth, horse serum (25%), and penicillin *G* for 7 days at 37°C. The concentration of *M. pneumoniae* was determined by 10^7^ color change units (CCUs)/ml.

### 2.2. Animals

Wild-type and TLR4-/- mice (C57BL/10ScNJ, 14–17 g, 3 weeks old) were obtained from the Laboratory Animals Center of Shanxi Medical University. All mice were maintained under the following conditions: 23 ± 2°C, 50 ± 10% humidity, and 12 h light-dark cycles, specific pathogen-free condition for a week, and free access to food and water. Mice were randomly divided into the control group (*n* = 5, administrated with 100 *μ*l normal saline). In *M*. *pneumoniae* group (*n* = 5), mice were intranasally infected with 100 *µ*l of *M*. *pneumoniae* solution (1 × 107 CCU/ml) once per day for two days as previously described [15]. Two days later, mice were anaesthetized with chloroform and sacrificed with cervical decapitation.

This study was approved by the Animal Care Board of Shanxi Provincial People's Hospital (SXPPH [2019]035).

### 2.3. HE Staining

The lower lobe of the right lung was fixed in 4% formaldehyde. Then, the sections were embedded with paraffin, dewaxed, dehydrated, and cultured with hematoxylin and eosin. Subsequently, sections were captured using Olympus microscopy (BX41-DP72) (×20).

### 2.4. Cell Treatment and Infection

Peritoneal macrophages RAW264.7 were exposed to 100 ng/ml LPS, 20 *μ*g TAK-242 (a TLR4 inhibitor, MCE, Shanghai), 30 *μ*M CCI-779 (a TFEB inhibitor, MCE, Shanghai), 40 µg chloroquine (CQ, Sigma-Aldrich, Shanghai), and 5 mM 3-methyladenine (3-MA, an autophagy inhibitor; Sigma-Aldrich). Next, the cells were infected with 0, 10, and 30 CFU/ml of *M*. *pneumoniae* for 24 h (OD595 = 0.1). The supernatants were harvested.

### 2.5. Enzyme-Linked Immunosorbent Assay (ELISA)

The levels of proinflammatory cytokines, such as TGF-*α* and IL-1*β*, were detected by ELISA kits (R&D, USA). Briefly, cells were plated into a 96-well plate (2 × 10^3^ cells/well) and incubated with biotinylated antibodies. Subsequently, the levels of TGF-*α* and IL-1*β* were determined with a microplate reader (ELx808, BioTeck, Shanghai) at the wavelength of 450 nm.

### 2.6. Cell Transfection

Small interference RNA TLR4 (5′-GGACCTCTCTCAGTGTCAA-3′) and its negative control (5′-ACUACUGAGUGACAGUAGA-3′) were provided by GenePharma, Shanghai. Cells were seeded into a 24-well plate (2 × 10^5^ cells/well) and were transfected with si-TLR4 and its negative control by using Lipofectamine® 2000 (Invitrogen, USA) according to the manufacturer's protocols for 48 h.

### 2.7. Western Blot

Total protein was collected from cells. Protein concentration was quantified using a BCA kit (Abcam, Shanghai). Afterwards, 30 µg of protein was separated by 12% SDS-PAGE at 120 V for 1 h. The separated protein was moved onto PVDF membranes (Millipore, Beijing), which was then sealed with nonfat milk. The membranes were incubated with primary antibodies including anti-TLR4 (ab13556, 1:500, Abcam, Shanghai), anti-TFEB (ab270604, 1:1000, Abcam, Shanghai), anti-LC3 I/II (ab128025, 1:1000, Abcam, Shanghai), anti-p62 (ab109012, 1:10000, Abcam, Shanghai), and anti-GAPDH (ab9485, 1:2500, Abcam, USA) at 4°C overnight and with secondary antibodies (ab205718, 1:10000, Abcam, Shanghai) at room temperature for 2 h. The bands were captured with an ECL kit (Abcam, Shanghai) and quantified using Scion Image v. 4.0.2 software (Scion Corporation).

### 2.8. Immunofluorescence Assay

Cells were seeded into a 24-well plate (2 × 10^3^ cells/plate). Then, cells were fixed and permeabilized. Cells were blocked with 2% bovine serum albumin in PBS for 30 min. After incubated with primary antibodies against TFEB (ab128025, 1:1000, Abcam, Shanghai) and LC3 puncta (ab192890, 1:1000, Abcam, Shanghai), cells were cultured with DAPI. Subsequently, the results were visualized with a confocal microscope (Zeiss, Germany).

### 2.9. Statistical Analysis

Data were analyzed with SPSS 19.0 and expressed as mean ± SD. The difference among multigroups was analyzed by ANOVA followed by Duncan's post-hoc test. *P* < 0.05 was considered statistically significant.

## 3. Results

### 3.1. TLR4-Deficient Mice Were Protected from *M*. *pneumoniae*-Induced Inflammatory Damage of Lung Tissues

As shown in Figures 1(a) and 1(b), lung structure was without any obvious lesion in TLR4-deficient mice. In *M*. *pneumoniae*-infected mice, the alveolar walls were thickened. Only a few bronchial tubes were narrowed, suggesting that TLR4 deficiency relieved inflammatory lung tissue damage after *M*. *pneumoniae* infection.

### 3.2. *M. pneumoniae* Induced the Secretion of IL-1*β* and TNF-*α* from Macrophages

*M. pneumoniae* promotes the inflammation response [7]. Macrophages were stimulated by LPS. ELISA was conducted to determine the levels of proinflammatory cytokines, including TNF-*α* and IL-1*β*. As shown in Figure 2(a), the level of TNF-*α* was significantly increased in cells exposed to LPS. Moreover, *M. pneumoniae* increased the level of TNF-*α* in a dose-dependent manner. This was paralleled with IL-1*β* (Figure 2(b)).

### 3.3. TLR4 Was Required for *M*. *pneumoniae*-Induced Inflammation in Macrophages

TLR4 is collectively involved in the progression of *M. pneumoniae* [13, 14]. As shown in Figures 3(a) and 3(b), *M. pneumoniae* infection further increased the expression of TLR4. To further verify this, cells were treated with si-TLR4. As shown in Figures 3(c) and 3(d), the protein expression of TLR4 was significantly decreased in cells transfected with si-TLR4, suggesting that cells were significantly transfected. Knockdown of TLR4 significantly inhibited the secretion of TNF-*α* and IL-1*β* (Figure 3(e)).

### 3.4. The Activation of TLR4 Promoted *M. pneumoniae*-Induced Inflammatory Response

Autophagy is reported to contribute to M. *pneumoniae* [4]. To further investigate the roles of autophagy in M. *pneumoniae*, immunofluorescence and western blot assays were applied to determine the expression of autophagic markers. As shown in Figure 4(a), the expression of LC3 puncta was significantly increased in cells treated with M. *pneumoniae*, which was alleviated by TAK-242. Moreover, *M. pneumoniae* upregulated LC3 II, Beclin-1, and Atg5 in a dose-dependent manner (Figures 4(b) and 4(c)). CQ treatment was to exclude the possibility that the upregulation of LC3 II was the result of LC3 II-induced lysosomal dysfunction. The ratios of LC3 II/I were decreased by *M*. *pneumoniae*, which was reversed by CQ (Figure 4(d)). However, *M*. pneumoniae-induced downregulation of p62 was alleviated by CQ (Figure 4(e)).

### 3.5. *M*. *pneumoniae*-Induced the Release of Proinflammatory Cytokines via Activating TFEB

TLR4 interacted with TFEB to modulate inflammation and autophagy [16, 17]. Therefore, we further investigated the potential roles of TFEB in *M*. pneumoniae-induced inflammation response, and macrophages were activated by *M. pneumoniae*. Immunofluorescence and western blot were conducted to determine the expression of TFEB. As shown in Figure 5(a), *M. pneumoniae* promoted the translocation of TFEB from the cytosol to the nucleus. Similarly, M. *pneumoniae* significantly upregulated TFEB, which was reversed by TAK-242 (Figures 5(b) and 5(c)). Moreover, *M. pneumoniae*-induced release of TNF-*α* and IL-1*β* was abated by TFEB inhibitor CCI-779 (Figures 5(d) and 5(e)).

Our work is to probe the impact of atorvastatin on rats during the retention stage after orthodontic tooth movement and its associated molecular mechanism, and to provide a theoretical basis and potential treatment for the relevant research and clinical treatment of orthodontic tooth retention and recovery.

### 3.6. TFEB Enhanced *M*. *pneumoniae*-Induced Autophagy

To further investigate the underlying molecular mechanisms in *M*. *pneumoniae*-induced autophagy, we investigate the potential roles. As shown in Figure 6(a), 3-MA alleviated the effects of *M*. *pneumoniae* on the translocation of TEBF from the nucleus was antagonized by 3-MA. Moreover, TFEB antagonist CCI-779 abated the effects of *M. pneumoniae* on the expression of LC3 puncta (Figure 6(b)–6(d)).

## 4. Discussion

Pulmonary lesions and metabolic disorders contribute to immune response and oxidative stress [4]. In this study, *M*. *pneumoniae* upregulated TLR4 and induced an inflammatory response. Downregulation of TLR4 inhibited inflammatory response and autophagy. Hence, TLR4 may play a crucial role in modulating autophagy and inflammatory response in *M*. *pneumoniae*.

TLRs recognize invading *M*. *pneumoniae* through interacting with its ligands such as LPS, FSL-1, lipoarabinomannan, and zymosan [9–11]. TLR4, an essential member of the TLRs family, promotes the development of *M*. *pneumoniae* via driving the secretion of lipid-associated membrane proteins, pulmonary inflammatory factors, cell apoptosis, and autophagy [18]. However, the potential roles of TLR4 in *M*. *pneumoniae* are alluring. LPS-activated TLR4 plays little role in *M. pneumoniae* recognition. However, Luo et al. reveal that activation induces inflammatory response and autophagy in M. *pneumoniae* [19].

TFEB, as a crucial member of MiT/TFE family, is a master of lysosomal-related processes including lysosomal exocytosis and autophagy [20]. Moreover, TFEB is an important player in innate and adaptive immunity [21]. The activation of TFEB in macrophages exposed to bacteria and various toll-like receptor (TLR) ligands contribute to innate immune response and pathogen resistance and the increase in autophagy that is an essential factor of HIV replication [22,23]. Moreover, the translocation of TFEB to nucleus promotes SARS 3a induced autophagy and necrotic cell death [24]. Hence, to inhibit lysosomal-related processes via suppressing the expression of TLR4/TFEB signaling may be an efficient therapy for the emerging innate immune response and pathogen resistance in *M*. *pneumoniae*.

Autophagy plays a crucial role in immune response induced by pathogenic micro-organisms [25]. The exacerbation of contributes to impairment of airway epithelial barrier and autophagy [4]. The activation of TLR4 pathways induces autophagy after *M. pneumoniae* infection [14]. In this study, knockdown of TLR4 suppressed the autophagy of RAW264.7. Moreover, chloroquine increased the expression of the autophagic adaptor protein expression of p62 and LC3 II, excluding possibility of decreased lysosomal fusion and degradation. Moreover, TFEB is the master regulator of autophagy signaling and links autophagy to lysosomal biogenesis [26]. Overexpression of TFEB predicts poor prognosis of non-small cell lung cancer [27]. TFEB-dependent autophagy induces the progression of emphysema [28]. In this study, TLR4/TFEB signaling participated in *M*. pneumoniae-induced inflammatory response and autophagy of macrophages. Knockdown of TLR4 suppressed the expression of TFEB and autophagy, which was alleviated by the inhibitor of TFEB (CCI-779). Therefore, TLR4/TFEB may play an essential role in *M. pneumoniae*-induced inflammation and autophagy. Moreover, recent studies reveal that SARS-CoV-2 takes advantage of the lysosomal/endosomal system to infect cells and that a paucity of SARS-CoV-2 infections among patients is followed in their Gaucher clinics (a type of lysosomes dysfunction) [29, 30]. Hence, to investigate the potential roles of TLR4/TFEB in *M*. *pneumoniae* infection may provide a potential strategy for COVID-19.

In conclusion, *M. pneumoniae* induced the activation of TLR4. TLR4 interacted with TFEB to form a positive feedback loop to promote inflammatory response and autophagy of macrophages. This may provide a novel strategy for treatment of *M*. *pneumoniae*.

## Figures and Tables

**Figure 1:** TLR4 deficiency abated *M. pneumoniae*-induced inflammatory damage of lung tissues. (a) HE staining was applied for histological analysis. Knockdown of TLR4 alleviated *M. pneumoniae*-induced inflammatory damage. (b) Quantification analysis of *A*^*∗∗*^*P* < 0.01, ^##^*P* < 0.01.

**Figure 2:** *M. pneumoniae*-induced the secretion of IL-1*β* and TNF-*α* from macrophages. (a) The level of IL-1*β* detected by ELISA. *M. pneumoniae* increased the levels of IL-1*β*. (b) The level of TNF-*α* detected by ELISA. *M. pneumoniae* increased the levels of TNF-*α*. *∗P* < 0.05, *∗∗P* < 0.01.

**Figure 3:** TLR4 promoted *M. pneumoniae*-induced proinflammation. (a) The protein expression of TLR4 detected by western blot. *M*. *pneumoniae* increased the protein of TLR4. (b) Quantification of A. (c) The protein expression of TLR4 detected by western blot. TLR4 was downregulated by si-TLR4. (d) Quantification of C (e) The levels of IL-1*β* and TNF-*α*. Knockdown of TLR4 decreased the levels of IL-1*β* and TNF-*α*. ^*∗∗*^*P* < 0.01, ##*P* < 0.01.

**Figure 4:** Autophagy promoted *M. pneumoniae*-induced inflammatory response. (a)The expression of LC3 II detected by immunofluorescence. Knockdown of TLR4 suppressed the upregulation of LC3 puncta induced by *M*. *pneumoniae*. (b)Quantification of A. (c) The protein expression of LC3 II/I, Beclin-1, and ULK1 determined by western blot. The protein expression of LC3 II/I and p62 increased the protein expression of LC3 II/I, Beclin-1, and ULK1. (d) Quantification of C. (e) The protein expression of LC3 II/I and p62 measured by western blot. *M. pneumoniae* increased the expression of LC3 II/I and p62, which was modulated by CQ. (f, g) Quantification of E. ^*∗*^*P* < 0.01, ^##^*P* < 0.01.

**Figure 5:** TFEB participated in *M. pneumoniae*-induced inflammatory response. (a)The expression of TFEB detected by immunofluorescence assay. *M. pneumoniae* increased the translocation of TFEB from the cytosol to the nucleus, which was reversed by TLR4 knockdown. (b) Quantification of A (c) The protein expression of TFEB determined by western blot. (d) Quantification of C. (e) The level of IL-1*β* and TNF-*α*. Knockdown of TFEB decreased the level of IL-1*β* and TNF-*α*. ^*∗∗*^*P* < 0.01, ^##^*P* < 0.01.

**Figure 6:** TFEB promoted *M. pneumoniae*-induced autophagy. (a) The expression of LC3 II detected by immunofluorescence. 3-MA suppressed the upregulation of LC3 puncta induced by *M. pneumoniae*. (b) Quantification of A. (c) The protein expression detected by western blot. Downregulation of TFEB reversed the increase of LC3 II induced by *M. pneumoniae.* (d) Quantification of C. (e) The expression of LC3 II detected by immunofluorescence. TFEB knockdown suppressed the upregulation of LC3 II induced by *M. pneumoniae*. ^*∗∗*^*P* < 0.01, ^##^*P* < 0.01.

## Data Availability

The experimental data used to support the findings of this study are available from the corresponding author upon request.
